This article has been retracted.

# Application of Nanocomposite Energy Storage Materials in Green Building Design

**DOI:** 10.1155/2022/7739734

**Published:** 2022-09-27

**Authors:** Ying Xu

**Affiliations:** Department of Architecture Engineering, Shijiazhuang Vocational Technology Institute, Shijiazhuang, Hebei 050000, China

## Abstract

In order to solve the problem of the application of composite phase change heat storage materials in building energy conservation, the author proposes the application of nanocomposite energy storage materials in green building design. Modified carbon nanotubes were prepared by mixed acid oxidation and ball milling, and composited with stearic acid to prepare phase change heat storage materials. Modified carbon nanotubes were prepared by mixed acid oxidation and ball milling and composited with stearic acid to prepare phase change heat storage materials. Experimental results show that acidified carbon nanotubes have a hindering effect on the thermal diffusion of stearic acid molecular segments so that the thermal conductivity of carbon nanotubes added with a mass fraction of 1% is only 1.3 times higher than that of pure stearic acid. *Conclusion*. Nanocomposite energy storage materials have excellent application prospects in green building design.

## 1. Introduction

Human activities are accompanied by the consumption of various energy sources, and energy problems have gradually become the main factor restricting regional development [1, 2]. However, the total energy consumption of various buildings is increasing year by year and building energy conservation and emission reduction have gradually become a new topic. With the development of green buildings from concept to practice, more and more new building energy-saving materials and technologies are being tried in buildings, such as solar energy technology, thermal insulation materials, and waste heat recovery technology.

As a kind of energy storage material, phase change material can realize energy exchange with the outside world through its own phase change process [3, 4]. When the external temperature decreases, the phase-change material can release the energy stored in the molecules, while maintaining itself within the phase change temperature range. When the ambient temperature increases, the external energy can be absorbed by the phase change material in large quantities and stored in the molecules of the phase change material, in this state, the phase change material is always in the phase change process and can maintain its own energy for a long time, the temperature does not change. Especially in the building environment, when the external environment temperature increases, the phase change material absorbs heat through the phase change process, so that the internal environment temperature is maintained within the comfort range of the human body.

Phase change materials are generally divided into inorganic and organic phase change materials. Inorganic phase change materials have the characteristics of large latent heat and strong heat transfer ability. But its defects are large phase transition undercooling and phase stratification phenomenon [5,6]. Contrary to the properties of inorganic phase change materials, organic phase change materials hardly have the disadvantages of phase change supercooling and phase stratification, and they have better durability, such as phase change paraffin, fatty acids, and some sterol materials. However, the latent heat of phase change of organic phase change materials is relatively low, and it is easy to cause environmental hazards. Most organic phase change materials are polymer materials with extremely high flammability, which limits their large-scale application in buildings. With the continuous and rapid development of the economy and industry, the energy crisis and greenhouse gas emissions are becoming more and more serious, and the efficient utilization and sustainable development of energy have become one of the urgent tasks faced by mankind. Thermal energy is a widely existing energy source in nature and a by-product of many energy conversion applications, energy storage is the recovery of abundant thermal energy, which can solve the contradiction between energy supply and demand in time and space and is a potential way to improve energy utilization efficiency. Therefore, developing new energy storage technologies and building efficient energy storage devices are considered to be one of the most effective strategies to save energy and protect the environment, as shown in Figure 1.

## 2. Literature Review

Phase change energy storage can alleviate the mismatch between energy supply and demand in terms of time, intensity, and location. It is an important technical means to improve energy utilization efficiency and energy conservation and emission reduction, and its research has attracted the attention of many scholars [7, 8]. With the continuous increase of population and the substantial growth of urbanized residents, the energy consumption of residential and commercial buildings accounts for a large part of my country's energy consumption. Therefore, combining the heat storage/release properties of phase change materials (PCMs) and applying them to the architectural field, is of great significance to alleviate the high energy consumption of buildings and the consequent environmental pollution problems.

With the continuous deepening of the idea of sustainable development, the problems of energy consumption and construction material pollution in the construction industry have been paid attention to. The government has promulgated relevant energy-saving and emission-reduction systems, and the construction industry must also comply with energy-saving emission reduction standards. When choosing construction raw materials, try to choose green and energy-saving materials, and choose renewable energy from limited resources and renewable energy. Although the cost may increase, it meets the requirements of sustainable development of the construction industry and is conducive to the development of environmental protection. The choice of new building materials is crucial, and building professionals are committed to researching the use of composite phase change heat storage materials. The composite phase change heat storage material is an energy-saving and environmentally friendly thermal insulation material, the heat storage function is realized by the energy change in the phase change, and the energy in the phase change material can be evenly distributed in the building wall to play the role of thermal insulation [9, 10]. With the growth of the population, the area of housing is also increasing, so the energy consumption of buildings is regulated, and the importance of energy saving is gradually spreading in the construction industry. The composite phase change heat storage material is not only green and environmentally friendly, but also has a good thermal insulation effect, the traditional thermal insulation material will cause solid waste pollution, and the thermal insulation effect is not as good as that of the composite phase change thermal storage material. When designing the wall, increasing the thickness of the construction can play a role in thermal insulation, and the cost of the thickened wall is higher. The thermal insulation principle of the composite phase change heat storage material is to store the external temperature for thermal insulation of the building. Phase change materials have the advantages of high density, easy temperature control, and the advantage of adjustable temperature and are widely used in the ever-developing smart building technology.

In this study, carbon nanotubes were modified by mixed acid oxidation and ball milling methods, the dispersibility was compared and a new composite phase change heat storage material was prepared by compounding with stearic acid. Test and characterize the thermophysical properties of composite phase change heat storage materials and study the nonisothermal phase change kinetic process of composite phase change heat storage materials, in order to reveal the microscopic kinetic mechanism of the effect of acidified carbon nanotubes on the thermophysical properties of stearic acid. The stearic acid/carbon nanotube composite phase change heat storage material can realize efficient heat utilization and storage and has important potential utilization for solar energy utilization.

## 3. Methods

### 3.1. Experimental Raw Materials and Experimental Equipment

The main raw materials of the experiment are multiwalled carbon nanotubes (CNT, outer diameter 10–20 nm, length 10–30 *μ*m, purity>95%, a nanomaterial technology Co., Ltd.), stearic acid (C_18_H_36_O_2_, SA), sulfuric acid (H_2_SO_4_, content 95%–98%), nitric acid (HNO_3_, content 65%–68%), etc., are all purchased from a group chemical reagent Co., Ltd. The experimental materials were used without any purification.

The main instruments and equipment of the experiment are precision electronic balance (JA2003, a scientific instrument Co., Ltd.), ultrasonic cleaning machine (KX-1613T, a century technology co., LTD.), collecting type constant temperature heating magnetic stirrer (DF-101S, an instrument, and equipment limited liability company), scanning electron microscope (JSM5610LV, Japan Electronics Co., Ltd.), X-ray diffractometer (D8 Advance, Bruker, Germany), Fourier transform infrared spectrometer (Nexus, Thermo Nicholas, USA), power-compensated differential scanning calorimeter (Pyris DSC, American PE company), and thermal constant analyzer (TPS 2500S, Sweden Hot Disk company).

### 3.2. Preparation of Stearic Acid/Carbon Nanotube Composite Phase Change Heat Storage Material

Acidification of carbon nanotubes is carried out as follows: weigh 1.0 g of carbon nanotubes and put them into a beaker with distilled water for 2 h ultrasonic dispersion. During this period, the beaker was taken out and cooled for 1 min every 15 min, and stirred with a glass rod, so that the carbon nanotubes were uniformly dispersed in the distilled water. Then, the dispersed carbon nanotubes were mixed with 40 mL of mixed acid (sulfuric acid/nitric acid volume ratio of 3 : 1) and placed in a water bath at 90°C for heating and magnetic stirring for 8 h. The obtained mixture was cooled to room temperature, washed with water until neutral, and placed in an oven at 60°C for 24 h to obtain the product, namely acidified carbon nanotubes (A-CNT).

Ball Milling of Carbon Nanotubes is carried out as follows: according to m_ball_:*m*_*CNT*_=200, put it into a ball milling jar, mill it for 720 min, wash it with water, and put it in a drying oven at 60°C for 24 h to obtain ball milled carbon nanotubes (B-CNT).

Preparation of composite phase change heat storage material is carried out as follows: the preparation of stearic acid (SA)/carbon nanotube (CNT) composite phase change heat storage material adopts a common melt blending method. After 0.1 g of carbon nanotubes were dispersed in the ethanol solution and sonicated for 0.5 h, they were added to 9.9 g of stearic acid that had been heated to complete melting in a water bath at 90°C and magnetically stirred for 1 h. The mixed sample was cooled to room temperature, the composite phase-change heat storage material (SA/CNT) with a mass fraction of carbon nanotubes of 1% was obtained, and its morphology, microstructure, thermophysical properties, etc., were characterized after grinding. The same procedure was used to prepare SA/A-CNT and SA/B-CNT with a mass fraction of 1%.

### 3.3. Material Phase and Microstructure

Figure 2 is the XRD patterns of CNTs, A-CNTs, and B-CNTs. Carbon nanotubes have strong diffraction peaks at 26.2° and 43.1°, which are their characteristic peaks. The carbon nanotubes treated with mixed acid did not generate new diffraction peaks, and the characteristic diffraction peaks did not shift, indicating that the phase of carbon nanotubes did not change after mixed acid oxidation. The diffraction peak of ball-milled carbon nanotubes has a small shift at 42.5° because the carbon nanotubes are broken, bent, and kinked by the impact during the ball-milling process, and the structure is damaged and structural defects are formed. But its physical phase did not change.

The unmodified carbon nanotubes have more impurity peaks in Figure 3. There are various synthesis methods for carbon nanotubes, but no matter which method is used to prepare carbon nanotubes, there are inevitably impurities such as catalysts, amorphous carbon, and graphite particles. Oxidation with mixed acid can remove some impurities and purify carbon nanotubes. The impurities present in the original carbon nanotubes are mainly particulate impurities such as amorphous carbon and carbon nanoparticles, during the acid treatment process, amorphous carbon is most easily oxidized, followed by carbon nanoparticles, while tubular carbon nanotubes can stablize their existence under conditions [11, 12]. This is mainly due to the multilayer structure of amorphous carbon, there are more dangling bonds at the edges, and the energy is high, so redox reactions are easy to occur. The carbon nanoparticles have a polyhedral structure with larger curvature and more five-membered rings, so they have higher reactivity. The oxygen-containing functional groups on the surface of the sample after mixed acid oxidation are assigned as follows: the high wavenumber bands at 3450 cm^−1^ and 3410 cm^−1^ can be assigned to the O–H stretching vibrations of carboxyl, phenolic, and hydroxyl groups on the CNT surface. The 1715 cm^−1^, 1580 cm^−1^, and 1500 cm^−1^ bands may be due to the *C*=*O* stretching vibration in the carboxyl group, lactone-type carboxyl group or carboxylic acid anhydride, ester, and other functional groups on the CNT surface, the 1210 cm^−1^ and 1120 cm^−1^ bands can then be assigned to the C–O stretching vibrations in the above-mentioned related oxygen-containing groups. The mixed acid oxidation changes the surface structure of the carbon nanotubes so that the surface of the carbon tube has carboxyl and hydroxyl functional groups, which increases the negative charge on the surface, the electrostatic repulsion between carbon tubes is enhanced, and the strong electrostatic repulsion makes the dispersion of carbon nanotubes in the solution more uniform, and it is not easy to form large agglomerates with each other, which improves their dispersibility in the solute.

### 3.4. Material Morphology

The entangled and agglomerated phenomenon of carbon nanotubes without any treatment is serious. After treatment, the surface of carbon nanotubes is relatively clean, the adhesion phenomenon disappears, the tube bundles are clear, and the dispersibility is good. Most of the tips and surfaces of carbon nanotubes have been covered with stearic acid. In appearance, carbon nanotubes cross each other, but because they are single tubes, the effective contact area between the tubes is not very large, and the reason why the stearic acid covers the surface and the tip makes the effective contact area between the tubes smaller. After ball milling, the agglomeration of CNTs was improved, and the dispersibility in stearic acid was significantly increased compared with untreated CNTs. However, after oxidative modification with mixed acid, the dispersibility of carbon nanotubes in stearic acid is the best, there is no obvious agglomeration phenomenon, and it is completely covered by stearic acid [13, 14].

### 3.5. Thermal Properties and Kinetics of SA/A-CNT Phase Change Heat Storage Materials

The modification of carbon nanotubes with high thermal conductivity is to improve the thermal conductivity of stearic acid by making them uniformly dispersed.  Table 1 is the thermal conductivity of stearic acid and its complexes. Adding carbon nanotubes did increase the thermal conductivity of stearic acid but not as well. The thermal conductivity of modified carbon nanotubes to stearic acid increases greatly. The effect of adding carbon nanotubes on the thermal conductivity of stearic acid is SA/A-CNT > SA/B-CNT > SA/CNT > SA, respectively. The thermal conductivity of acidified carbon nanotubes to stearic acid is increased by 1.3 times. It shows that mixed acid oxidation can effectively disperse the agglomeration of carbon nanotubes.

Figures 3 and 4 show the DSC curves of SA/A-CNT at different heating rates. The heating rates *β*=5*C* · min^−1^, 10*C* · min^−1^, 15*C* · min^−1^, and 20C · min^−1^, are shown in Figures 4 and 5. With the increase of the heating rate, the peak shape of the heating DSC curve of SA/A-CNT is shifted to the right, and the peak temperature is shifted to the high-temperature direction, and the temperature range of the phase transition reaction became wider. Because the heating rate is high, the SA molecular chain has no time to diffuse out of the crystal.

The Kissinger approximation equation for nonisothermal phase transition kinetics is as follows:

(1) $$\begin{array}{c} \ln\frac{\beta }{T_{p}^{2}}=C-\frac{E}{RT_{p}}, \end{array}$$

in(*β*/*T*_*p*_^2^) and 1/*T*_p_ have a linear relationship, the corresponding intercept, slope, and correlation coefficient (*r*) can be obtained from the linear regression calculation of the peak temperature *T*_p_ at different heating rates *β* , and the activation energy *E* of the melting process can be obtained from the slope.

## 4. Results and Discussion

Figure 6 shows the linear fitting curves of ln(*β*/*T*_*p*_^2^) and 1000/*T*_*p*_ of SA/A-CNT and pure SA obtained by the Kissinger kinetic method [15,16]. The regression curve of pure SA is *y*=319.22 − 113.30*x*, the slope is −*E*/*R*=−113.30, and the activation energy *E*=941.98kJ · mol^−1^ of pure SA is calculated. The regression curve is *y*=339.55 − 120.06*x*, the slope is −*E*/*R*=−120.06, and the activation energy *E*=998.18*kJ* · *mol*^−1^ can be calculated. From the activation energy obtained from the slope of the straight line in Figure 6, it can be seen that the activation energy of SA/A-CNT composite phase change heat storage material is higher than that of pure SA. Acidified carbon nanotubes have a limiting effect on the thermal diffusion of SA molecular segments, which increases the phase transition activation energy of SA/A-CNT composites and makes the phase transition process more difficult. This is also the reason why the thermal conductivity of SA/A-CNT is only 1.3 times higher than that of pure SA.

The apparent activation energy of the composite phase change heat storage material is higher than that of pure stearic acid, indicating that the acidified carbon nanotubes have a hindering effect on the thermal diffusion of stearic acid molecular segments, which increases the difficulty of the phase change process and affects the hardness of the stearic acid, the increase of the thermal conductivity of stearic acid increases the thermal conductivity by only 1.3 times that of pure stearic acid after adding 1% mass fraction of carbon nanotubes [17, 18]. The X-ray diffraction results showed that the ball milling treatment had a certain influence on the structure of carbon nanotubes, and the phase of carbon nanotubes after mixed acid oxidation did not change. Infrared spectrum analysis showed that ball milling and mixed acid oxidation could purify carbon nanotubes, and functional groups such as hydroxyl and carbonyl appeared in acidified carbon nanotubes, which were helpful for the dispersion of carbon nanotubes. Scanning electron microscope pictures show that the dispersibility of modified carbon nanotubes in stearic acid is acidified carbon nanotubes > ball-milled carbon nanotubes > carbon nanotubes [19, 20].

## 5. Conclusion

The author proposes the application of nanocomposite energy storage materials in green building design. Compared with ball milling, mixed acid oxidation has less damage to the structure of carbon nanotubes, and the surface and ports of the acidified carbon nanotubes produce active groups such as hydroxyl and carboxyl groups, which increase the repulsive force between the carbon tubes, reduce the van der Waals force, and increase the distance between the tube walls and increase the affinity between carbon nanotubes and solute. So, the phenomenon of entanglement and agglomeration between acidified carbon nanotubes is reduced, and the dispersion in stearic acid is more uniform, which is conducive to heat transfer.

## Figures and Tables

**Figure 1:** Guidelines for green building design.

**Figure 2:** XRD patterns of CNT, A-CNT, and B-CNT.

**Figure 3:** Infrared spectra of CNT, A-CNT, and B-CNT.

**Figure 4:** DSC curves of pure SA at different heating rates.

**Figure 5:** DSC curves of SA/A-CNT at different heating rates.

**Figure 6:** Kissinger curves of SA/A-CNT and SA.

**Table 1:** Thermal conductivity of stearic acid and its composite phase change heat storage materials, unit: W/(m.K).

Sample	SA	SA/CNT	SA/B-CNT	SA/A-CNT
Thermal conductivity	0.33	0.35	0.40	0.43

## Data Availability

The data used to support the findings of this study are available from the corresponding author upon request.
